# Bioinformatics Analysis for Identifying Pertinent Pathways and Genes in Sepsis

**DOI:** 10.1155/2021/2085173

**Published:** 2021-11-01

**Authors:** Yiran Li, Hongyan Zhang, Jinyan Shao, Jindong Chen, Tiancheng Zhang, Xiaoyan Meng, Ruiqing Zong, Guangzhi Jin, Feixiang Wu

**Affiliations:** ^1^Department of Intensive Care Medicine, Eastern Hepatobiliary Surgery Hospital, Second Military Medical University, Shanghai, China; ^2^Department of Emergency, Minhang Hospital, Fudan University, China; ^3^School of Basic Medical Sciences, The Second Military Medical University, Shanghai, China; ^4^Medical College of Soochow University, Soochow University, 199 Renai Road, Suzhou 215123, China; ^5^Department of Anesthesiology, Tongren Hospital, Shanghai Jiao Tong University School of Medicine, 1111 Xianxia Road, Shanghai 200336, China

## Abstract

**Purpose:**

Sepsis becomes the main death reason in hospitals with rising incidence, causing a growing economic and medical burden. However, the genes related to the pathogenesis and prognosis of sepsis are still unclear, which is a problem that needs to be solved urgently.

**Materials and Methods:**

Gene expression profiles of GSE69528 were obtained from the National Center for Biotechnology Information. Limma software package got employed to search for differentially expressed genes (DEGs). Kyoto Encyclopedia of Genes and Genomes (KEGG) and Gene Ontology (GO) were used for enrichment analysis. Protein-protein interaction (PPI) network was built by the Search Tool for the Retrieval of Interacting Genes (STRING) database.

**Results:**

We screened 101 DEGs, containing 81 upregulated DEGs and 20 downregulated DEGs. GO analysis demonstrated that the upregulated DEGs were chiefly concentrated in negative regulation of response to interferon-gamma and regulation of granulocyte differentiation. KEGG analysis revealed that the pathways of upregulated DEGs were concentrated in prion diseases, complement and coagulation cascades, and Staphylococcus aureus infection. The PPI network constructed by upregulated DEGs contained 67 nodes (proteins) and 110 edges (interactions). Analysis of bioinformatics results showed that CEACAM8, MPO, and RETN were hub genes of sepsis.

**Conclusion:**

Our analysis reveals a series of signal pathways and key genes related to the mechanism of sepsis, which are promising biotargets and biomarkers of sepsis.

## 1. Background

Sepsis is a serious syndrome characterized by infection changes in physiology, pathology, and biochemical life [1]. It has become a main death reason for hospital deaths in intensive care unit (ICU) patients and millions of deaths worldwide every year [2]. In the United States, 10% of ICU patients have sepsis, and about 25% of ICU beds are occupied by sick patients [3]. The updated sepsis-3 criteria record sepsis as a severe organ dysfunction because of patients' dysfunctional responses to infection [4]. The advancement of medicine career has increased the rate of survivors after primary sepsis injury. Acute death is not the main reason for sepsis death. Nowadays, 70% of sepsis-related deaths happen in the first three days after its onset, which is caused by secondary infection [5].

The pathogenesis of sepsis is very complicated and currently unclear, so the treatment of sepsis is limited [6]. The mechanisms include systemic inflammation, coagulation, fibrinolytic disorders, and excessive production of reactive oxygen and nitrogen [6]. Sepsis becomes the main reason for severe patients' death. There are currently no specific therapeutic drugs approved for the treatment of sepsis, and treatment options are limited [7]. Sinha et al. point out that despite advances in molecular diagnostic technology, blood culture analysis is still the gold standard for the diagnosis of sepsis [8]. At present, these molecular technologies have been verified on clinical blood samples or simulated samples using human blood.

Bioinformatics plays a key role in supporting life sciences and brings unique opportunities and challenges to human disease research [9]. Based on bioinformatics analysis, it is found that the long noncoding RNA LINC00426 is downregulated in the tumor tissues of NSCLC patients, which is associated with poor prognosis [10]. A new oncogene VPS35 was identified in hepatocellular carcinoma by DNA and RNA sequencing [11]. This study analyzes the gene expression profile GSE69528 and screens DEGs related to sepsis through a series of biological information technologies. Finally, the key pathways and genes are obtained. CEACAM8, MPO, and RETN have the potential to become key biotargets for sepsis.

## 2. Materials and Methods

### 2.1. Microarray Data

Microarray data were acquired from Gene Expression Omnibus (GEO), an accessible functional genomics database of high-throughput resources, which was one of the most commonly used sequencing (chip) databases in the National Center for Biotechnology Information (NCBI) (https://pubmed.ncbi.nlm.nih.gov/). The microarray data set GSE69528 was downloaded from Illumina HumanHT-12 V4.0 expression beadchip in the GEO database. The whole RNA of blood from sepsis patients caused by Pseudomonas (*n* = 29) or other pathogens (*n* = 28) and uninfected controls (28 healthy people) were collected from GSE69528.

### 2.2. Differentially Expressed Genes (DEGs) Identification

The original data of mRNA expression profile were downloaded and delved by the R language software. The genes whose *P* value < 0.01 and fold change (FC) > 3/2 or FC < 2/3 were regarded as DEGs. Then, the researchers used the heat map package in R to construct a heat map. The heat map shows data in a two-dimensional form, in which colors represent the values, providing an instant visual overview of the information. More sophisticated heat maps help observers understand complex data sets.

### 2.3. Gene Ontology (GO) and Kyoto Encyclopedia of Genes and Genomes (KEGG) Analysis

GO (http://www.geneontology.org.) [12] is the result of efforts to make the functional description of gene products in various databases consistent. KEGG (http://www.genome.jp/kegg/) [13] is a knowledge base analyzing gene function systems that connect genomic information and high-level functional information. For the enrichment analysis of GO and KEGG, we used Database for Annotation, Visualization and Integrated Discovery (DAVID) (https://david.ncifcrf.gov/tools.jsp) for processing.

### 2.4. Protein-Protein Interaction (PPI) Network Construction of DEGs

The Search Tool for the Retrieval of Interacting Genes (STRING) (http://string-db.org) is a database for searching interactions between proteins. It includes both the direct physical interaction and the indirect functional correlation between proteins. When the interaction score > 0.4, it is considered significant. STRING got utilized to build a PPI network. The purpose was to find out the hub genes related to sepsis.

### 2.5. Statistical Analysis

The R software was used for the statistical analysis of DEGs. We used *t*-test or Mann–Whitney *U* test to make statistical comparisons of standardized data sets. *P* less than 0.05 meant that there was a significant difference in compared groups.

## 3. Result

### 3.1. Identification of DEGs in Sepsis

To study the hub genes and pathways in sepsis, the whole RNA of blood from sepsis patients caused by Pseudomonas (*n* = 29) or other pathogens (*n* = 28) and uninfected controls (28 healthy people) were collected from the gene expression profile GSE69528. The heat map was utilized to analyze the cluster analysis of the identified DEG in the GSE69528 database (Figure 1). On the basis of the standard of *P* < 0.01 and fold change (FC) > 3/2 or FC < 2/3, we screened 101 DEGs, including 81 upregulated genes and 20 downregulated genes.

### 3.2. GO and KEGG Enrichment Analysis of DEGs in Sepsis

Through DAVID online database enrichment analysis, we found that the biological processes (BPs) of upregulated DEGs were majorly enriched in negative regulation of response to interferon-gamma, negative regulation of interferon-gamma-mediated signaling pathway, and regulation of granulocyte differentiation (Figure 2). The KEGG pathways of upregulated DEGs were mainly enriched in prion diseases, complement and coagulation cascades, and Staphylococcus aureus infection (Figure 3).

### 3.3. PPI Network Construction

The screened upregulated DEGs were subsequently used to construct the PPI network through the STRING database. The PPI network was comprised of 67 nodes (proteins) and 110 edges (interactions) (Figure 4). The screening of hub genes adopted the degree analysis method in Cytoscape. The higher the degree, the more closely the gene was associated with sepsis. The results illustrated that the degree of CEACAM8 was 17, MPO was 12, and RETN was 10. We could summarize that CEACAM8, MPO, and RETN are hub genes of sepsis. CEACAM8, MPO, and RETN were significantly upregulated in sepsis (Figure 5).

## 4. Discussion

Sepsis becomes the main reason for severe patients' death [14]. In the United States, 1 to 3 million patients are infected with sepsis each year, resulting in 250,000 to 350,000 deaths in hospitals [15]. As the pathogenesis and treatment methods are still unclear, the clinical treatment of sepsis has brought a great burden to society and patients [16]. Looking for potential biomarkers is important for future sepsis treatment and prognosis. A systematic review by Tang et al. shows that the host response of sepsis is not in line with a simple high-inflammation/low-inflammation model [17]. Therefore, we synthesize the current genomic study to examine the host's response to human sepsis in circulating white blood cells. Qiu et al. point out that molecular hydrogen has anti-inflammatory, antioxidant, antiapoptotic, antishock, autophagy, and other biological effects and could reduce organ and barrier damage caused by sepsis [18]. Mathias et al. mention that granulocyte-macrophage colony-stimulating factor (GM-CSF) is a hematopoietic growth factor currently used in patients with neutropenia caused by chemotherapeutic myelosuppression, which could combat the immunosuppression of sepsis period [19].

Our research results found that negative regulation of response to interferon-gamma and regulation of granulocyte differentiation were the top significant enriched BPs of upregulated DEGs. And prion diseases, complement and coagulation cascades, and Staphylococcus aureus infection were the top significant enriched KEGG pathways of upregulated DEGs. Cirulis et al. propose that interferon is a cytokine that stimulates innate and adaptive immune responses and involved in the early proinflammatory and delayed immunosuppressive stages of sepsis [20]. Staphylococcus aureus is a gram-positive pathogen that colonizes human skin and nostrils and the main cause of soft tissue infection and bacterial sepsis in humans [21]. Inhibiting the growth of Staphylococcus aureus and improving the body's immune mechanism are of far-reaching significance for the control and treatment of sepsis.

Through the use of STRING online database and Cytoscape processing tools for analysis, we found that the gene most associated with sepsis is CEACAM8, MPO, and RETN. Jog et al. propose that CEACAM 8 belongs to the carcinoembryonic antigen (CEA) family of the immunoglobulin superfamily [22]. CEAMs participate in a variety of intercellular adhesion and cell signal-mediated effects and regulate immune responses related to pathogen binding, inflammation, and the growth and/or differentiation of normal cells and cancer cells [23]. In recent years, researchers have found that when sepsis occurs, the concentration of extracellular chromatin increases, and extracellular chromatin triggers the release of soluble CEACAM 8 during the activation of neutrophils, and CEACAM8 exerts an immunomodulatory effect [4, 24]. As we all know, MPO is an indicator of neutrophil infiltration as well as the severity of inflammation during sepsis [25]. At the same time, MPO is the main enzyme produced by neutrophils and has an antibacterial function in sepsis [26]. Demaret et al. believe that in patients with sepsis, reduced MPO expression is considered to be the best predictor for identifying the subgroup of high-risk death patients, and treatment can reduce MPO expression, thereby reducing oxidative stress damage in sepsis [27]. Resistin (RETN) is an adipocyte-specific hormone secreted by WAT3 [28]. It is also a key mediator of immunosuppression [29]. Immunosuppression is critical to the morbidity and mortality associated with sepsis [30]. Therefore, controlling the secretion of RETN has special meaning for sepsis treatment.

This study has some limitations. First, the expression level of key genes needs to be verified by qRT-PCR. Secondly, the specific mechanism of the hub gene in sepsis needs to be further explored. In future studies, we will collect enough clinical samples to further explore the correlation between the expression of CEACAM8, MPO, and RETN and the prognosis of patients with sepsis.

## 5. Conclusion

In a word, we screened 101 DEGs from sepsis patients caused by B. pseudomallei (*n* = 29) or other pathogens (*n* = 28) and uninfected controls (*n* = 28). According to the screening, 81 upregulated DEGs and 20 downregulated DEGs got obtained. Negative regulation of response to interferon-gamma and regulation of granulocyte differentiation are the main biological processes. Prion diseases, complement and coagulation cascades, and Staphylococcus aureus infection are the most critical signaling pathways. Finally, through the analysis of the PPI network, we discover hub genes related to sepsis: CEACAM8, MPO, and RETN. These pathways and genes provide research directions for sepsis initiation and progression and may participate in sepsis future research.

## Figures and Tables

**Figure 1:** Heat map analysis of identified DEGs between patients with sepsis caused by B. pseudomallei or other pathogens and uninfected controls. The red color shows the upregulated DEGs, and the blue color is the downregulated DEGs.

**Figure 2:** Biological process analysis of upregulated DEGs in sepsis patients.

**Figure 3:** KEGG analysis of upregulated DEGs in sepsis patients.

**Figure 4:** The PPI networks were established by significant upregulated DEGs which contain 67 nodes and 110 edges. Nodes mean proteins, and edges mean the interaction of proteins.

**Figure 5:** The expression level analysis of CEACAM8, MPO, and RETN according to GSE69528 database.

## Data Availability

The datasets used and/or analyzed during the current study are available from the corresponding author on reasonable request.
